The article "Clinical Application of Remifentanil Combined with Sevoflurane in Manual Reduction of Humeral Supracondylar Fracture in Children" was retracted in 2023. Reasons: signs of a paper mill; suspected computer-generated content; unreliable results or conclusions; concerns about the data.

# Clinical Application of Remifentanil Combined with Sevoflurane in Manual Reduction of Humeral Supracondylar Fracture in Children

**DOI:** 10.1155/2022/2410433

**Published:** 2022-07-08

**Authors:** Youqing Li, Jiangping Yu, Mingmin Zhang, Meng Jia

**Affiliations:** Department of Anesthesiology, Hangzhou Fuyang Hospital of Orthopedics of Traditional Chinese Medicine, Fuyang, Zhejiang 311400, China

## Abstract

**Objective:**

To explore the effect of the combination of remifentanil and sevoflurane on children with humeral supracondylar fractures undergoing manual reduction.

**Methods:**

A total of 60 children undergoing manual reduction external fixation due to humeral supracondylar fractures were enrolled between September 2020 and September 2021. According to the random number table method, they were divided into the control group (inhalation of 7% sevoflurane) and the observation group (inhalation of 7% sevoflurane and intravenous infusion of remifentanil). The heart rate (HR), mean arterial pressure (MAP), and blood oxygen saturation (SpO_2_) in both groups were investigated. The sedation and analgesic effects, fracture reduction, and complications were compared between the two groups.

**Results:**

There was no significant difference found in HR, MAP, or SpO_2_ between the two groups at 3 minutes prior to anesthesia, 2 minutes post anesthesia, and post manual reduction (*P* > 0.05). The difference in HR, MAP, and SpO_2_ between the two groups was not statistically significant at any time point (*P* > 0.05). The good rate of sedation and analgesia in the observation group was 93.33%, which is significantly higher than that in the control group (*P* < 0.05). The reduction time and success rate of one-time manual reduction in the observation group were higher than those in the control group (*P* < 0.05). There was no significant difference in fracture healing time between the two groups (*P* > 0.05). Both groups had airway complications (nausea and vomiting, neurovascular damage and asphyxia, and laryngospasm).

**Conclusion:**

The combination of remifentanil and sevoflurane showed good sedative and analgesic effects on children with humeral supracondylar fractures undergoing manual reduction with relatively higher safety.

## 1. Introduction

Children are prone to accidental fractures, especially supracondylar fractures of the humerus, in daily life. Therapeutic treatments such as manual reduction and external fixation are effective for some children [1]. Specifically, manual reduction under conventional brachial plexus anesthesia is proven to be an outstanding treatment method for children. However, due to the low cooperation of children during brachial plexus anesthesia, general compound anesthesia is often needed. Prolonged general compound anesthesia duration makes it less favorite for operation [2]. Sevoflurane, a new type of inhaled anesthetic, has no pungent smell, light inhibition of respiration and circulation, fast induction, and quick and complete recovery, resulting in its increasing use in child anesthesia induction [3]. However, sevoflurane does not show a good analgesic effect. During manual reduction, the body movement of children caused by body pain could increase the difficulty of manual reduction and the risk of anesthesia [4]. Remifentanil is the first ultrashort effect opioid used in general anesthesia with rapid onset and short duration. It has been widely used in children's surgical anesthesia with the trend of solid controllability, rapid onset, and continuous use [5]. Furthermore, the combination of remifentanil and sevoflurane showed a good anesthetic effect on various short and minor operations [6, 7]. However, the actual effect of the above combination is not fully evaluated. Thus, this study is aimed at investigating the effect of the combination of remifentanil and sevoflurane on the manual reduction of supracondylar fracture of humerus in children. This study could provide guidelines on future operations and thus increase the comfortability of medical treatment for kids.

The article "Clinical Application of Remifentanil Combined with Sevoflurane in Manual Reduction of Humeral Supracondylar Fracture in Children" was retracted in 2023. Reasons: signs of a paper mill; suspected computer-generated content; unreliable results or conclusions; concerns about the data.

## 2. Methods

### 2.1. General Information

60 children with a humeral supracondylar fracture who underwent manual reduction and external fixation from September 2020 to September 2021 were randomly divided into the control group (only inhaled 7% sevoflurane) and the observation group (inhaled 7% sevoflurane+intravenous infusion of remifentanil), with 30 cases in each group. All general information is collected in Table 1. There is no significant difference found in age, sex ratio, and ASA grade between the two groups (*P* > 0.05). This study was in line with the declaration of Helsinki, and the families of the children signed informed consent.

### 2.2. Inclusion and Exclusion Criteria

Inclusion criteria include the following: (1) the child was diagnosed with a supracondylar fracture of humerus by clinical physical examination and X-ray examination [8], (2) age is between 4 and 10 years, (3) ASA was classified as grade I~II, and (4) family members voluntarily received manual reduction treatment.

Exclusion criteria include the following: (1) patients with neuromuscular diseases; (2) patients with a previous history of heart disease or bronchial asthma; (3) patients with severe liver, kidney, and coagulation dysfunction; (4) patients with allergy to drugs included in the study; and (5) family members who refused to participate in the study or were unable to cooperate.

The article "Clinical Application of Remifentanil Combined with Sevoflurane in Manual Reduction of Humeral Supracondylar Fracture in Children" was retracted in 2023. Reasons: signs of a paper mill; suspected computer-generated content; unreliable results or conclusions; concerns about the data.

### 2.3. Intervention Methods

Atropine sulphate injection (Jiangsu Lianshui Pharmaceutical Co., Ltd., national drug approval H32020166, specification: 1 mL: 0.5 mg) of 0.01 mg/kg was administrated in both groups 30 min prior to operation. The venous channel was opened, and ECG, blood oxygen saturation (SpO_2_), and blood pressure were monitored after entering the room. The children in the control group were provided with an oxygen flow of 6 L/min and 7% sevoflurane (Shanghai Hengrui Pharmaceutical Co., Ltd., national drug approval H20070172, specification: 120 mL). Children retained spontaneous breathing and were given manual assistance if necessary. The observation group was also given sevoflurane inhalation. After the eyelash reflex disappeared, the children in the observation group were given intravenous remifentanil hydrochloride injection (Jiangsu Enhua Pharmaceutical Co., Ltd., national drug approval H20143314, specification: 1 mg) of 0.15 *μ*g/(kg·min); manual reduction and external fixation were performed 2 minutes later. The manual reduction in both groups was performed by the same physician. After manual reduction, intraoperative C-arm fluoroscopy was used to determine the fracture reduction and external fixation with a fir bark splint.

### 2.4. Observation Index

The heart rate (HR), mean arterial pressure (MAP), and blood oxygen saturation (SpO_2_) of the two groups were recorded 3 min prior to anesthesia, 2 min post anesthesia, and post manual reduction. The sedative and analgesic effects, fracture reduction (reduction time, fracture healing time, and success rate of one-time manual reduction), and complications (nausea and vomiting, vascular and nerve injury, airway complications, etc.) were compared. The criteria for determining the sedative and analgesic effects [9] were excellent (no pain and limb movement during operation, quick awakening after operation, and no bad memory), good (slight limb twisting during operation, unconscious groaning, acceptable awake quality after operation, and no bad memory), and poor (children are restless during operation, feel severe pain after waking up, and have bad memory).

### 2.5. Statistical Method

Statistical software SPSS19.0 was used to analyze and process data. Measurement data confirming normal distribution was expressed as the mean ± standard deviation, and Student's *t*-test was used to compare the two means. The counting data were expressed in percentage (%). The *χ*^2^ test was used for nonranked data, and the Ridit test was used for ranked data. *P* < 0.05 indicated that the difference was statistically significant.

The article "Clinical Application of Remifentanil Combined with Sevoflurane in Manual Reduction of Humeral Supracondylar Fracture in Children" was retracted in 2023. Reasons: signs of a paper mill; suspected computer-generated content; unreliable results or conclusions; concerns about the data.

## 3. Results

### 3.1. Comparison of Changes in HR, MAP, and SpO_2_ between the Two Groups

There was no significant difference in HR, MAP, and SpO_2_ between the two groups 3 min prior to anesthesia, 2 min post anesthesia, and post manual reduction (*P* > 0.05). The statistical evaluation is summarized in Table 2.

### 3.2. Comparison of Sedative and Analgesic Effects between the Two Groups

The sedative and analgesic effects of the observation group were better than that of the control group. As shown in Table 3 and Figure 1, the difference was counted as statistically significant.

### 3.3. Comparison of Fracture Reduction between the Two Groups

The reduction time of the observation group was shorter than that of the control group, and the difference was statistically significant (*P* < 0.05). There was no significant difference in the fracture healing time between the two groups (*P* > 0.05). The success rate of one-time manual reduction in the observation group was higher than that in the control group; however, the difference was not statistically significant (*P* < 0.05), as shown in Table 4.

### 3.4. Comparison of Complications between the Two Groups

There were no airway complications such as nausea and vomiting, vascular and nerve injury, asphyxia, and laryngospasm in both groups.

## 4. Discussion

The direct impact is the leading cause of supramalleolar fracture of the humerus in children. Supposing the palm is directly supporting the body weight when falling, the elbow joints are put in the extended position, and the lower end of the humerus is directly taking the impact and thus resulting in supramalleolar fracture. As children's bones are in a relatively active state of growth and have strong shaping ability, after fracture, children can recover well through scientific exercise and reasonable fixation. Therefore, simple conservative treatment can be carried out if there is no displacement of humeral supramalleolar fracture in children [10]. In the past, manual reduction was operated without anesthesia. The difficulty of manual reduction was increased due to children's natural fear, sharp pain, and muscle tension during manual reduction, resulting in a low success rate of one-time reduction [11]. With the requirement of multiple manual reductions, consequences such as neurovascular injury are not conducive to fracture healing. The incompletion of manual reduction and surgical treatment could increase patients' dissatisfaction and further lead to medical disputes. Manual reduction anesthesia has high requirements for narcotic drugs, especially for children. Narcotic drugs need to take effect quickly, relieve pain quickly, reduce muscle tension, awake patients entirely and rapidly post operation, and cause a lower incidence of adverse reactions. At present, sevoflurane is often induced by inhalation through a mask, and it takes only 2 minutes to enter the anesthesia state [12]. Another drug, remifentanil, is an opioid *μ* receptor agonist with the characteristics of fast onset, short maintenance time, strong analgesic effect, and short half-life [13]. Ying [14] illustrated that remifentanil had an excellent analgesic effect on pediatric surgery without respiratory depression and low postoperative agitation and stress response incidence. Evaluating the drug characteristics of both remifentanil and sevoflurane, the combination of the two could possibly achieve rapid anesthesia induction and sufficient analgesia for children.

The article "Clinical Application of Remifentanil Combined with Sevoflurane in Manual Reduction of Humeral Supracondylar Fracture in Children" was retracted in 2023. Reasons: signs of a paper mill; suspected computer-generated content; unreliable results or conclusions; concerns about the data.

This study used remifentanil combined with sevoflurane for anesthesia induction in the manual reduction of humeral supracondylar fracture in children. It was found that there was no significant difference in HR, MAP, and SpO_2_ between the two groups 3 minutes prior to anesthesia, 2 minutes post anesthesia, and post manual reduction, suggesting that both combination of remifentanil and sevoflurane and sevoflurane alone had little effect on hemodynamics in children. The study has indicated that although remifentanil does not inhibit myocardial contractility, it could cause bradycardia [15]. In this study, the HR of children is only slightly reduced with no statistical difference. The results might be caused due to the fact that a low dose of remifentanil was not sufficient to cause respiratory depression. The sedative and analgesic effects of remifentanil combined with sevoflurane are better than that of sevoflurane alone, which is consistent with the results of previous studies [16], suggesting that the combination of remifentanil and sevoflurane could maintain an appropriate depth of anesthesia. At the same time, remifentanil also has the dual effects of sedation and analgesia. It has an immediate and strong effect that compensates sevoflurane anesthesia deficiency. In this study, the reduction time and the success rate of one-time manual reduction in the observation group were better than those in the control group, indicating that the effect of sevoflurane alone on manual reduction was mildly insufficient. With sevoflurane only, children exhibited limb activities due to pain, which increased the difficulty of operation, resulting in the extension of reduction time and decrease of the one-time manual reduction success rate. There is no significant difference in fracture healing time between the two groups. It is worth noting that manual reduction only needs to maintain the stability and rationality of fracture reduction to avoid overcorrection. In addition, vascular and nerve injuries and other complications were observed after reduction. Although the two groups of children had mild airway complications such as nausea and vomiting, vascular and nerve injury, asphyxia, and laryngeal spasm, no serious complications were observed, indicating that the two anesthesia methods were still with high safety capability.

The article "Clinical Application of Remifentanil Combined with Sevoflurane in Manual Reduction of Humeral Supracondylar Fracture in Children" was retracted in 2023. Reasons: signs of a paper mill; suspected computer-generated content; unreliable results or conclusions; concerns about the data.

In conclusion, the combination of remifentanil and sevoflurane showed good sedative and analgesic effects on the manual reduction of supracondylar humeral fractures in children. The vital signs of children during the operation were stable without serious complications, which will help improve the hospital's rapid recovery, painless, and comfortable medical services.

## Figures and Tables

**Figure 1:** Comparison of changes in HR, MAP, and SpO_2_ between the two groups.

**Table 1:** Comparison of the general conditions of the two groups of children.

	Control (*n* = 30)	Observation (*n* = 30)	*χ* ^2^/*t*	*P*
Gender (*n*, %)				
Male	21, 70.00	19, 63.33	0.3	0.584
Female	9, 30.00	11, 36.67		
Age (years)	6.87 ± 1.43	7.23 ± 1.25		
Hospital time (hours)	3.53 ± 1.11	3.67 ± 1.18	0.465	0.644
ASA classification (*n*)				
I	15	12	0.61	0.436
II	15	18		

**Table 2:** Comparison of changes in HR, MAP, and SpO_2_ between the two groups ($\bar{x}\pm s$, *n* = 30).

Group	Time	HR (beats/min)	MAP (mmHg)	SpO_2_ (%)
Control	3 min before anesthesia	105.12 ± 11.42	78.67 ± 8.54	98.40 ± 0.72
	2 min after anesthesia	84.73 ± 9.87	76.33 ± 8.14	98.60 ± 0.72
	Manual reduction	85.13 ± 10.56	75.53 ± 8.29	98.80 ± 0.61
	After waking up	92.23 ± 8.14	75.87 ± 8.06	99.03 ± 0.32

Observation	3 min before anesthesia	100.23 ± 10.59	79.13 ± 8.87	98.73 ± 0.45
	2 min after anesthesia	84.38 ± 10.25	76.93 ± 8.23	98.50 ± 0.63
	Manual reduction	86.53 ± 11.24	75.20 ± 8.06	98.83 ± 0.46
	After waking up	93.43 ± 9.66	76.00 ± 7.96	98.93 ± 0.45

**Table 3:** Comparison of sedative and analgesic effects between the two groups (*n* (%)).

Group	Excellent	Good	Poor
Control	10 (33.33)	12 (40.00)	8 (26.67)
Observation	19 (63.33)	9 (30.00)	2 (6.67)
*U*			2.51
*P*			0.012

**Table 4:** Comparison of fracture reduction between the two groups (score).

Group	Reset time (min)	Fracture healing time (day)	Success rate of one-time manual reduction (*n* (%))
Control	15.53 ± 4.23	41.37 ± 4.39	24 (80.00)
Observation	11.97 ± 2.68^∗^	40.50 ± 5.62	29 (96.67)
*χ* ^2^/*t*	3.894	0.668	2.59^∗^
*P*	<0.001	0.507	0.108

^∗^Adopted Yates-corrected chi-squared test.

## Data Availability

The labeled dataset used to support the findings of this study is available from the corresponding author upon request.
